# Diagnosis of Atherosclerotic Plaques Using Vascular Endothelial Growth Factor Receptor-2 Targeting Antibody Nano-microbubble as Ultrasound Contrast Agent

This article has been retracted.

**DOI:** 10.1155/2022/6524592

**Published:** 2022-05-05

**Authors:** Yi Wang, Yujin Feng, Xiaoyun Yang, Wengang Wang, Yueheng Wang

**Affiliations:** Department of Ultrasonography, The Second Hospital of Hebei Medical University, Shijiazhuang, 050000 Hebei, China

## Abstract

The atherosclerotic plaque is characterized by narrowing of blood vessels and reduced blood flow leading to the insufficient blood supply to the brain. The hemodynamic changes caused by arterial stenosis increase the shearing force of the fibrous cap on the surface of the plaque, thereby reducing the stability of the plaque. Unstable plaques are more likely to promote angiogenesis and increase the risk of patients with cerebrovascular diseases. A timely understanding of the formation and stability of the arterial plaque can guide in taking targeted measures for reducing the risk of acute stroke in patients. It has been confirmed that nano-microbubbles can enter these plaques through the gaps in the patient's vascular endothelial cells, thereby enhancing the acquisition of ultrasound information for plaque visualization. Therefore, we aim to investigate the diagnostic value of targeted nano-microbubbles for atherosclerotic plaques. This study constructed vascular endothelial growth factor receptor-2 (VEGFR-2) targeting antibody nano-microbubbles and compared its diagnostic value with that of blank nano-microbubbles for atherosclerotic plaques. Studies have found that VEGFR-2 targeting antibody nano-microbubbles can accurately detect the position of plaques. Its detection rate, sensitivity, and specificity for plaques are higher than those of blank nano-microbubbles. Similarly, the peak intensity and average transit time of VEGFR-2 targeting antibody nano-microbubbles were greater than those of blank nano-microbubbles. Therefore, we believe that the combination of VEGFR-2 antibody and nano-microbubbles can enhance the acquisition of ultrasound information on atherosclerotic plaque neovascularization, thereby improving the early diagnosis of unstable plaque.

## 1. Introduction

Atherosclerotic plaque, a specific manifestation of atherosclerosis, is considered to be the main cause of ischemic stroke and acute cerebral infarction in patients. It poses a serious threat in patients with atherosclerosis [1]. Arteriosclerotic plaque generally occurs at the site of bifurcation of the common artery, mainly due to arterial lipid deposition. The resulting plaques can narrow blood vessels and reduce blood flow, leading to the insufficient blood supply to the brain [2]. The hemodynamic changes caused by arterial stenosis increase the shearing force of the fibrous cap on the surface of the plaque, which reduces the stability of the plaque [3]. Unstable plaques are also referred to as vulnerable plaques. This type of plaque is more likely to promote regeneration of blood vessels and increase cerebrovascular disease risk in patients. Therefore, timely understanding of arterial plaque formation in patients plays an important role in deciding targeted measures to reduce the risk of acute stroke in patients. The pathological examination results are considered to be the gold standard for clinical identification of the vulnerability of the plaque. However, the process of pathological examination is traumatic and has certain limitations in the early diagnosis. As a commonly used clinical diagnostic method, ultrasound can accurately detect the location of arterial stenosis in a comparatively shorter time span, which is of great significance for assessing atherosclerotic plaque [4, 5]. Traditional ultrasound mainly produces images based on the characteristics of the difference in propagation speeds of sound waves between different tissues. Medical professionals diagnose diseases based on the characteristics of these resulting images. Recently, there has been rapid development in the ultrasound technology, and contrast-enhanced ultrasound technology has been widely used clinically. Common contrast-enhanced ultrasound technologies include hysterography, breast ultrasound contrast, and liver ultrasound contrast [6–8]. However, traditional contrast agents can only diagnose diseases at a macrolevel through enhanced organ imaging and still lack the ability to reflect the characteristics of the disease at the microlevel. As a result, the development of targeted ultrasound contrast agents that can reflect the microscopic diseases of the organs for diagnosis has become a research hotspot.

An ultrasound microbubble contrast agent is a liquid solution containing bubbles with a diameter between 1 and 8 *μ*m, which are injected into human blood vessels to enhance the ultrasound signal of blood flow, thereby improving the clarity and resolution of resulting ultrasound images [9, 10]. Due to the limited flexibility of human blood cells and the ability of microbubbles to increase the spacing between human tissues, the microbubbles can enhance ultrasound signals. At the same time, the air bubbles provide an enhanced imaging effect, which helps to determine the regularity of the plaque surface or bleeding. Although conventional microbubbles can enhance the image effect, they are limited by their diameter and cannot penetrate the vascular endothelium [11]. The nano-microbubbles are approximately 500 nm in diameter, which enables them to enter the plaque through the gaps in the patient's vascular endothelial cells, thereby enhancing the acquisition of ultrasound information for plaque visualization [12]. With the continuous development of ultrasound microbubble contrast agents, clinical research on nanoscale ultrasound microbubbles has made great progress. Some scholars have reported that the goal of targeted therapy can be achieved through nano-microbubbles carrying drugs with therapeutic effects and their controlled release in designated areas [13]. Also, nano-microbubbles are not easily cleared by the reticuloendothelial system due to their special properties. Therefore, nano-microbubbles have a longer circulation time as compared to that of traditional ultrasound microbubbles in the patient's body, thereby improving the utilization of therapeutic agents [14]. Due to the abovementioned characteristics, nanoscale ultrasound microbubbles have become the current focus of ultrasound imaging research. However, recent studies have found that it is not the degree of vascular lumen stenosis, but the morphology and composition of arteriosclerotic plaque that are the main factors causing acute clinical symptoms in patients [15, 16]. The primary pathological feature of atherosclerotic plaque is the generation of a large number of blood vessels in the plaque.

Therefore, we aim to construct a targeted ultrasound contrast agent with specific diagnostic and therapeutic effects and provide a reference for the diagnosis and treatment of plaque with drug-loaded ultrasound nano-microbubble contrast agents. We integrated vascular endothelial growth factor receptor-2 (VEGFR-2) with nanoscale ultrasound microbubbles.

## 2. Materials and Methods

### 2.1. Animals, Reagents, and Instruments

Sixty healthy 12-month-old Sprague Dawley rats (240−270 g) were provided by Guangxi Animal Experimental Center (the methods and purposes of animal experiments conform to human moral and ethical standards and international practices). DSPE-PEG2000 was provided by Lipoid, Ludwigshafen, Germany. Soybean phospholipids were provided by Shanghai Fetal Pharmaceutical Co., Ltd. Tween-80 and 1,2-dimyristoyl-sn-glycero-3-phosphocholine (DMPC), VEGFR-2 antibody, fluorescein isothiocyanate (FITC), and streptavidin were procured from Hubei Zhongliao Chemical Co., Ltd.; Avanti, USA; CST, Germany; Beijing Zhongshan Jinqiao Company; and Thermo Fisher, USA, respectively. The cell crusher; high-speed centrifuge; transmission electron microscope; fluorescence microscope; and color doppler ultrasound system were procured from Shanghai Xiyang Instrument Co., Ltd.; Shanghai Jingsheng Scientific Instrument Co., Ltd.; Thermo Fisher Scientific; Olympus, Japan; and Jiangsu Dawei Medical Co., Ltd.

### 2.2. Animal Model Preparation

The rats were fed a high-fat diet for a period of two months. This high-fat diet was prepared by adding 5% lard and 0.5% cholesterol to the basic feed. The aim of this high-fat diet was to cause damage to their vascular endothelium. The rats were allowed to perform normal activities and have regular water intake during this period.

### 2.3. Preparation of Nano-Microbubbles Loaded with VEGFR-2 Antibody

The selection of appropriate biomarkers is a crucial factor for the success of targeted microbubble technology since it has a huge impact on the clarity, sensitivity, and specificity of ultrasound imaging. VEGFR-2 is a receptor protein of vascular endothelial growth factor. It is highly expressed in the endothelial cells of unstable plaque neovascularization.

In order to prepare the blank nano-microbubbles (nanoscale lipid microbubbles), 0.02 g DSPE-PEG2000 and 0.1 g soybean phospholipids were dissolved in 20 mL normal saline (containing 1% Tween-80) and then added 0.4 g DMPS. The obtained solution was placed in a cell pulverizer for ultrasonic emulsification (the emulsification time was set to 2 min), and sulfur hexachloride gas (SF6) was continuously introduced during emulsification process. The emulsified nano-microbubbles were stored at 4 °C for 5 h. After the nano-microbubbles were naturally stratified, the upper layer containing microbubbles with a larger diameter was discarded. The lower layer of the solution was collected and resuspended to obtain the nano-microbubbles of appropriate diameter.

To prepare nano-microbubbles loaded with targeting VEGFR-2 antibody, streptavidin was added to the abovementioned blank nano-microbubbles. These nano-microbubbles were incubated at 25 °C for 1 h followed by centrifugation and washing to obtain avidin-biotinylated microvesicles. Biotinylated VEGFR-2 antibody was added to the obtained microvesicles and incubated for 12 h at 25 °C. Lastly, mix with fluorescein isothiocyanate– (FITC–) labeled biotin-labeled goat anti-mouse IgG diluent (1 : 4,000). The mixed solution was incubated at 37 °C for 1 h to obtain fluorescent-labeled VEGFR-2 targeted ultrasonic nano-microbubbles. A transmission electron microscope was used to observe the morphology and distribution of the prepared nano-microbubbles. The particle size distribution and average particle size of the nano-microbubbles were detected using a laser particle size analyzer.

### 2.4. *In Vivo* Contrast-Enhanced Ultrasound Analysis

The ultrasound contrast agent is a chemical agent that enhances ultrasound echo by improving the intensity of ultrasound backscatter, thereby displaying the size and position of blood vessels more clearly in ultrasound diagnosis. Although the use of ultrasound contrast agents was initially limited to ultrasound diagnosis, it has been extended to ultrasound therapy in recent years.

The sixty rats were randomly divided into two equal groups. After weighing routinely, anesthetizing, and preparing the skin, the rats were fixed on the operating table in a supine position. Nano-microbubbles were injected through the tail vein at the concentration of 0.5 mL/kg body weight. The pipe was flushed with normal saline after injection with a contrast medium. A color ultrasound diagnostic apparatus was used to detect the arteries of rats. The probe was set to the normal contrast mode and the frequency was set to 4 MHz.

Regular calcification (vascular remodeling and plaque formation), calcified plaque (hemorrhage in the plaque and neovascularization), mixed plaques (visible bright yellow plaques in the blood vessels), lipid plaques (nodular calcification on the surface of the plaques), and ulcerative plaques (the distance between adjacent plaques exceeds 0.2 mm, and there is vascular endothelium) are the five known types of plaque types and contrast-enhanced ultrasound diagnostic criteria [17]. The occurrence of one or more of the above five types of plaque is suspected as the presence of arteriosclerotic plaque. After the ultrasound examination, the lesion tissue of the experimental rat was dissected by surgery, and pathological examination was performed. The pathological examination result was used as the gold standard for comparison of the detection value of the two kinds of nano-microbubbles to plaque. At the same time, the detection time-intensity curve changes of the two types of nano-microbubbles were compared.

### 2.5. Statistical Analysis

In this study, Statistical program for Social Sciences (SPSS) v.25.0 and GraphPad Prism v.8.2 software was used for data analysis. Quantitative data are expressed as mean ± standard deviation. Comparisons between two groups, multiple groups, and pairwise comparisons between multiple groups were performed by Student's *t-*test, analysis of variance, and SNA-Q test, respectively. Qualitative data are represented by *n* (%), and the chi-square test was also performed. *P* < 0.05 indicates that the difference is significant for respective data comparisons.

## 3. Results

### 3.1. Observation of Nano-microbubble Morphology

Through transmission electron microscopy, the VEGFR-2 targeting nano-microbubbles were seen as uniformly distributed with good dispersibility (Figure 1(a)). Nano-microbubbles with a diameter less than 700 nm passed through the vascular endothelial space. Here, the laser particle size analyzer revealed that the prepared VEGFR-2 targeted nano-microbubbles had an average particle size of 423.76 ± 67.59 nm (Figure 1(b)). This suggests that the VEGFR-2 targeting nano-microbubbles prepared in this study meet the requirements of atherosclerotic plaque ultrasound contrast agents.

### 3.2. Observation of Fluorescent Labeling of Nano-microbubbles

Observation of the dispersion of FITC-labeled nano-microbubbles using a fluorescence microscope revealed an excellent dispersion of nano-microbubbles (Figure 2). The surface of the nano-microbubbles is visible as a bright circular fluorescence in the fluorescence imaging mode. No other fluorescence exists except for the background of the nano-microbubbles. This suggests that the VEGFR-2 antibody successfully binds to the microvesicles.

### 3.3. *In Vivo* Ultrasound Imaging

Rats injected with blank nano-microbubbles showed thickening of blood vessels when observed using *in vivo* imaging (the red circle in Figure 3(a)). The internal and external areas of the blood vessel and the vessel wall were also observed. However, more accurate positioning could not be achieved. Observation of the rats injected with VEGFR-2 targeted nano-microbubbles revealed that the echo between the tissues was significantly enhanced, the plaque was clearly distinguished from the surrounding tissues (the red circle in Figure 3(b)), and the location of the plaque could be determined. The above results suggest that VEGFR-2 targeting nano-microbubbles can enhance the effect of ultrasound contrast imaging and targeting.

### 3.4. Comparison of Time-Intensity Related Parameters Using Different Contrast Media

Ultrasound observation of the rats injected with ultrasound nano-microbubbles through the tail vein showed that most arterial plaques were rich in blood supply. Analysis of the time to peak (TTP), peak intensity (PI), and mean transit time (MTT) values for the two groups revealed that the PI and MTT of the VEGFR-2 group were significantly higher than those of the blank group (*P* < 0.05) (Table 1 and Figure 4).

### 3.5. Value Comparison of Different Nano-microbubbles in Plaque Detection

Comparing the diagnostic value obtained from pathological examination of the two kinds of nano-microbubbles on atherosclerotic plaques revealed that the detection rate of VEGFR-2 targeting nano-microbubbles on atherosclerotic plaques in rats was higher than that of blank nano-microbubbles. Similarly, the sensitivity and specificity of VEGFR-2 targeting nano-microbubbles for detecting atherosclerotic plaques were also higher than that of blank microbubbles (Table 2 and Figure 5).

## 4. Discussion

Atherosclerosis and its related complications are the main causes of mortality in patients with cardiovascular diseases. Previous studies reported that it was a series of clinical symptoms following vascular stenosis caused by hardened plaque. Therefore, the degree of luminal stenosis in patients is clinically regarded as an essential basis for the selection of clinical treatment options and prognosis [18]. However, the number and distribution of these newly developed blood vessels are not only the main factors affecting the stability of the plaque, but also the main cause of acute cardiovascular symptoms in patients [19]. Therefore, early understanding of the formation and distribution of plaque neovascularization and taking corresponding measures is required to mitigate the risk of an acute ischemic syndrome caused by plaque rupture.

The main component of clinically used ultrasound contrast agents is a microbubble enveloping a gas or liquid. Microbubbles can easily circulate through the patient's lungs to enhance visualization of its cavitation, thereby enhancing the acquisition of ultrasound information for biological entities [20]. With the expansion of the use of ultrasound contrast agents, their application value in many aspects, such as ultrasound thrombolysis, drug delivery, mediating gene transfer, and ultrasound high-intensity focused therapy, has also been continuously improved [21–23]. Targeted ultrasound contrast agents connect specific antibodies to the surface of microbubbles and bind to specific antigens in the patient's body through the antibodies, thereby enhancing the resulting echo of the target tissue [24]. Therefore, targeted contrast agents carrying specific ligands have good development prospects in the detection of plaque stability. Targeted microbubbles loaded with drugs can not only achieve specific treatment of targeted tissues and organs, but also reduce the damage caused by drugs to nontargeted tissues and organs.

VEGFR-2 antibody, a targeted ultrasound microbubble carrying biomarker, has become a research hotspot [25]. Liu et al. reported that the retention rate of targeted contrast agents in plaques was significantly higher than that of nontargeted plaques, suggesting that targeted contrast agents can improve ultrasound imaging clarity of plaques [26]. Baron Toaldo et al. have also confirmed through research that VEGFR-2 targeting microbubbles can improve the early evaluation of liver cancer by ultrasound imaging [27]. In this light, we prepared nanoscale lipid microbubbles and confirmed their dispersing ability by observing them under transmission microscope. The laser particle size analyzer found that the diameter of the microbubbles was 423.76 ± 67.59 nm, which fully met the particle size requirements of ultrasound contrast agents for atherosclerotic plaques. The VEGFR-2 antibody was further combined with nano-microbubbles, and the combined rate of the two was found to exceed 80% by flow cytometry. Diagnosis of atherosclerotic plaques using VEGFR-2 targeting nano-microbubbles contrast agent revealed that the diagnostic detection rate, sensitivity, and specificity of VEGFR-2 targeting nano-microbubbles were improved as compared to the corresponding values recorded using blank nano-microbubbles. The rate of misdiagnosis was also reduced in case of VEGFR-2 targeting nano-microbubbles. The time-intensity curve change objectively reflects the characteristics of the time-varying contrast medium perfusion in the plaque. When comparing the time-intensity curve changes of the two types of nano-microbubbles, it was found that the PI and MTT of the VEGFR-2 targeted nano-microbubbles were greatly higher than the blank nano-microbubbles. The above results suggest that VEGFR-2 targeting nano-microbubbles can enhance the acquisition of ultrasound information for atherosclerotic plaques. Comparing the diagnostic value of the two nano-microbubbles for atherosclerotic plaque, it was seen that the VEGFR-2 targeting antibody nano-microbubble accurately located the position of the plaque, and its detection rate, sensitivity, and specificity were higher than the blank nano-microbubbles. Comparing the time-intensity curve changes for the two kinds of nano-microbubbles, it was found that the PI and average transit time of the VEGFR-2 targeting antibody nano-microbubbles were greatly higher than the blank nano-microbubbles.

## 5. Conclusion

In summary, we constructed VEGFR-2 targeting antibody nano-microbubbles and confirmed their dispersing ability by observing them under a transmission electron microscope. The laser particle size analyzer confirmed that the average particle size of the VEGFR-2 targeting antibody nano-microbubbles met the size requirements of atherosclerotic plaque ultrasound contrast agent. The surface of nano-microbubbles illuminated as a bright circular structure when observed under a fluorescence microscope, thereby indicating that the VEGFR-2 antibody successfully binds specifically to the microvesicles. It was proved that the combination of VEGFR-2 antibody and nano-microbubbles enhances the acquisition of ultrasound information on atherosclerotic plaque neovascularization, thereby improving the diagnosis of early unstable plaque.

## Figures and Tables

**Figure 1:** Morphological observation and particle size analysis of VEGFR-2 (a) targeted nano-microbubbles. Transmission electron microscopic observation of VEGFR-2 targeting nano-microbubbles. (b) The particle size distribution of VEGFR-2 targeting nano-microbubbles.

**Figure 2:** Observation of the fluorescent labeling of VEGFR-2 targeted nano-microbubbles. (a) VEGFR-2 targeting nano-microbubbles in optical imaging mode. (b) VEGFR-2 targeting nano-microbubbles in fluorescence imaging mode.

**Figure 3:** *In vivo* imaging of two types of microbubbles. (a) Imaging effect of blank nano-microbubbles. (b) Imaging effect of VEGFR-2 targeting nano-microbubbles.

**Figure 4:** Comparison of the time-intensity-related parameters under different contrast media. The comparison of two types of nano-microbubbles for (a) time to peak (TTP), (b) peak intensity (PI), and (c) mean transit time (MTT).

**Figure 5:** Comparison of the detection values of different nano-microbubbles for plaque.

**Table 1:** Comparison of the time-intensity related parameters under different contrast media.

Groups	Time to peak (s)	Peak intensity (%)	Mean transit time (s)
VEGFR-2	24.85 ± 4.67	63.85 ± 10.29	31.08 ± 5.68
Blank	24.62 ± 4.19	31.52 ± 9.44	24.33 ± 5.09
t	0.087	6.946	2.655
*P*	0.931	<0.001	0.017

**Table 2:** Comparison of the detection values of different nano-microbubbles for plaque.

Groups	Relevance ratio	Sensitivity	Specificity
VEGFR-2	96.67 (29/30)	85.00 (16/20)	88.89 (8/9)
Blank	90.00 (27/30)	73.68 (14/19)	75.00 (6/8)
t	1.071	0.219	0.562
*P*	0.301	0.640	0.453

## Data Availability

The fingerprint data used to support the findings of this study are available from the corresponding author upon request.
